The article "Renal Denervation Mitigated Fecal Microbiota Aberrations in Rats with Chronic Heart Failure" was published in 2021. Journal: Evid Based Complement Alternat Med.

# Renal Denervation Mitigated Fecal Microbiota Aberrations in Rats with Chronic Heart Failure

**DOI:** 10.1155/2021/1697004

**Published:** 2021-10-15

**Authors:** Zhiqin Guo, Yufeng Chen, Shuoxian Chen, Chao Liu, Shaonan Li, Pingan Chen

**Affiliations:** ^1^Department of Cardiology, The Second Affiliated Hospital, School of Medicine, South China University of Technology, Guangzhou, China; ^2^School of Basic Medical Sciences, Qiqihar Medical University, Qiqihaer, China; ^3^Department of Electrocardiogram, Guangzhou First People's Hospital, School of Medicine, South China University of Technology, Guangzhou, China

## Abstract

**Background:**

Changes in the composition and diversity of gut microbiota, which can be altered by autonomic nerve activity, contribute to the development of heart failure (HF). Renal denervation (RDN) can improve cardiac function by reducing sympathetic nerve activity. However, whether the beneficial role of RDN on HF is related to gut microbiota is unknown.

**Methods:**

Thirty rats were assigned to a control, HF (with induced transverse aortic constriction (TAC)), RDN (with RDN induced 10 weeks after TAC), Nog (HF rats with Nogo-P4-administered 8 weeks after RDN), and NEP (HF rats with NEP1-40-administered 8 weeks after RDN) group. Then, 16SrRNA amplicon sequencing and analyses of fecal samples were performed.

**Results:**

Beta diversity analyses revealed that compared to the HF group, the RDN, Nog, and NEP groups clustered closer to the control group. The *Firmicutes*/*Bacteroidetes* ratio was reduced in the HF group (1.59) compared with the control group (3.21) and was significantly decreased compared to the Nog (7.19), RDN (6.20), and NEP (4.42) groups. At the genus level, the HF group showed decreased abundances of *Lactobacillus* and *Alistipes* and increased abundances of *Bacteroides* and *Clostridium* compared with the control group. The abundances of *Lactobacillus* and *Alistipes* were increased, and those of *Bacteroides* and *Clostridium* were decreased in the RDN, Nog, and NEP groups compared to the HF group. However, no differences were observed between the three groups that underwent RDN. The microbial function showed the same tendency.

**Conclusions:**

RDN reversed the abnormal changes in the gut microbiome in HF rats. Inhibition of reinnervation after RDN did not affect intestinal bacteria.

## 1. Introduction

Heart failure (HF) is a common, costly, and life-threatening disease [1]. Despite the availability of pharmacological approaches, the mortality of chronic heart failure remains high. Heart failure is a global pandemic due to its increasing prevalence and poor prognosis [2].

Altered gut microbiota is associated with several chronic diseases including HF. The severity and prognosis of HF can be influenced by gut bacteria and their products. Some special products of intestinal bacteria such as trimethylamine (TMA) [3] and butyrate [4] can affect cardiac function. Changes in the composition and diversity of the gut microbiome have also been observed in HF [5].

However, gut microbiota and their hosts' nervous systems are in constant communication via neural, endocrine, and immunological mechanisms [6]. Therefore, there is a connection between the gut microbiome and the sympathetic nervous system [7]. Increased sympathetic drive to the gut is associated with increased gut wall permeability, elevated inflammatory status, and microbial dysbiosis [8], and these gut pathological changes are linked to HF. Downregulation of pathological sympathetic activity is a key therapeutic strategy for HF [9–11]. Renal denervation (RDN) is an emerging therapeutic strategy for HF that results in the ablation of renal sympathetic nerve activity and further decreases global sympathetic tone [12]. Our previous study demonstrated that RDN improved cardiac function in dogs with HF [13]. However, few studies have focused on the relationship between RDN and intestinal bacteria in HF. Some studies have found functional reinnervation of the renal vasculature after RDN [14, 15], but whether this nerve regeneration affects gut microbiota or RDN efficacy is unknown.

We hypothesized that RDN could reverse intestinal microflora aberrations observed in HF rats and had a beneficial effect on cardiac function by influencing intestinal bacteria. Therefore, this study aimed to investigate the specific changes in gut microbiome composition and function in HF rats before and after RDN. We also explored the effects of regulating nerve regeneration after RDN on cardiac function and intestinal microbiota by intraperitoneally injecting Nogo-P4, an inhibitor of axonal regeneration [16], or NEP 1-40, a Nogo receptor competitive antagonist [17], into the rats.

## 2. Materials and Methods

### 2.1. Animals

A total of 30 SPF Sprague–Dawley rats (bodyweights 160–220 g for males and 100–150 g for females, 8 weeks old) purchased from Guangdong Medical Laboratory Animal Center were assigned into five groups as follows: (1) in the control group (*n* = 4), the rats received sham transverse aortic constriction (TAC), sham RDN, and an intraperitoneal injection of 2 ml of 0.9% saline; (2) in the HF group (*n* = 7), the rats received TAC to induce HF, sham RDN, and an intraperitoneal injection of 2 ml of 0.9% saline; (3) in the RDN group (*n* = 6), the rats received TAC, RDN 10 weeks after TAC, and an intraperitoneal injection of 2 ml of 0.9% saline; (4) in the Nog group (*n* = 7), the rats received TAC and RDN 10 weeks after TAC and were intraperitoneally injected with 0.02 mg (0.001%, 2 ml) Nogo-P4 (Alpha Diagnostics, San Antonio, TX, catalog no. Nogo-P4) daily for 2 weeks at 8 weeks after RDN; and (5) in NEP group (*n* = 6), the rats received TAC and RDN and were intraperitoneally injected with 0.025 mg (0.00125%, 2 ml) NEP 1–40 (APExBIO, Houston, TX, USA, Catalog No. B5247) daily for 2 weeks at 8 weeks after RDN (Figure 1(a)).

All the rats were housed in a clean environment under a 12-h light-dark cycle with free access to food and water. This investigation conforms to the *Guide for the Care and Use of Laboratory Animals* published by the US National Institutes of Health (NIH Publication No. 85-23, revised in 1985). The protocol was approved by the institutional ethics committee of Guangzhou First People's Hospital.

### 2.2. Establishment of the Heart Failure Model

Heart failure was induced by TAC. The rats were anesthetized with 2% pentobarbital sodium (30 mg/kg, intraperitoneally injected). The suprarenal abdominal aorta was exposed through a midline abdominal incision and isolated from the surrounding tissue. Abdominal aortic constriction was performed using a 4-0 suture tied around the suprarenal aorta and a blunt needle (23G), and then the needle was removed immediately. The rats were treated with penicillin and returned to their home cages after surgery. Sham-operated rats were subjected to the same surgeries except for ligation of the aorta.

### 2.3. Operation of Renal Denervation

After anesthetization with 2% pentobarbital sodium (30 mg/kg, intraperitoneally injected), the rats were placed in a supine position, and the left kidney was exposed by a median longitudinal incision. Unilateral left renal denervation was performed by stripping the renal artery and painting it with 10% phenol in absolute alcohol. Right renal denervation was performed in the same way. The muscle and skin layers were separately sutured. The rats were treated with antibiotics after surgery. Sham RDN rats were subjected to the same surgeries except for painting the left and right renal arteries with saline water.

### 2.4. Enzyme-Linked Immunosorbent Assay (ELISA)

In the 16th week after intraperitoneal administration, plasma N-terminal prohormone B-type natriuretic peptide (NT-proBNP) levels were measured using the NT-proBNP ELISA Kit (Wuhan CUSABIO Science Co. Ltd., China) according to the manufacturer's protocol.

### 2.5. Stool Sample Collection and DNA Extraction

In the 16th week after intraperitoneal administration, after blood collection, rats were sacrificed by pentobarbital sodium overdose (100 mg/kg). The intestines were dissected with sterile scissors, and the contents of the intestines were collected with a sterile device. Fresh stool samples from each group were immediately frozen in a liquid nitrogen tank and then stored at −80°C. The CTAB/SDS method was adopted to extract all of the genomic DNA from the samples, and the genomic DNA sample was diluted to 1 ng/*μ*l using sterile water. Moreover, fresh stool samples from the Con group (*n* = 5, rats that received sham RDN) and Con + RDN group (*n* = 5, rats that received RDN) were also collected.

### 2.6. Sequencing

16S rRNA sequencing was performed at the Novogene Bioinformatics Co. Ltd. (Tianjin, China). The V4 region of 16S rRNA genes was analyzed. The specific primers 515F (5′-GTGCCAGCMGCCGCGGTAA-3′) and 806R (5′-GGACTACHVGGGTWTCTAAT-3′) with the barcodes were applied to amplify 16S rRNA genes. An NEB Next®Ultra™ DNA Library Prep Kit for Illumina (NEB, USA) was used to produce sequencing libraries, and index codes were added. The library was sequenced on an Illumina MiSeq platform.

### 2.7. Data Analysis

The same operational taxonomic units (OTUs) consisted of sequences with a similarity of 97%. Alpha diversity was represented by the abundance coverage estimator (ACE) and observed species. Principal component analysis (PCA), principal coordinate analysis (PCoA) based on the unweighted UniFrac distance, and nonmetric multidimensional scaling (NMDS) were performed using R software to describe the beta diversity. To determine the differences in microbial communities between groups, analysis of similarity (ANOSIM), analysis of molecular variance (AMOVA), analysis of distance matrices (ADONIS), and MRPP (multiresponse permutation procedure) were carried out. The difference in individual taxonomy between groups was analyzed by Metastats (http://metastats.cbcb.umd.edu/) [18]. The biomarkers within different groups were quantitatively analyzed by linear discriminant analysis effect size (LEfse) [19]. Gut microbial functions were evaluated using the KEGG (Kyoto Encyclopedia of Genes and Genomes) database [20]. The experimental data were shown as the means ± standard deviation or median (lower quartile-upper quartile). *P* < 0.05 was considered to indicate a statistically significant result. Nonparametric tests and one-way ANOVA with LSD post hoc tests were used. Statistical analysis was performed using SPSS software (SPSS version 20.0).

## 3. Results

### 3.1. RDN Decreased Plasma NT-proBNP Levels in Rats with Heart Failure

As shown in Figure 1(b), the plasma levels of NT-proBNP were significantly higher in the HF rats than in the controls (218.46 ± 47.36 vs. 146.80 ± 12.14 pg/ml; *P*=0.006). Rats in the RDN group (155.98 ± 30.07 vs. 218.46 ± 47.36 pg/ml; *P*=0.016), the Nog group (130.64 ± 34.29 vs. 218.46 ± 47.36 pg/ml; *P*=0.002), and the NEP group (124.96 ± 18.29 vs. 218.46 ± 47.36 pg/ml; *P*=0.001) had significantly lower plasma NT‐proBNP levels than those in the HF group.

### 3.2. There Was No Significant Difference in Alpha Diversity between the Five Groups

Amplicon sequencing technology was used to sequence the 16S rDNA of the gut flora of rats from 30 samples from 5 groups. An average of 78,210 sequences per sample was obtained. These sequences were clustered into 2,747 OTUs at a 97% similarity threshold.

The rarefaction curves gradually tended to be flat with the increased number of sequences. This meant that even if the sequencing depth was expanded, no more bacterial species were detected. The rarefaction curves showed that the data volume of this study was reasonable, and the sequencing depth was sufficient, meeting the requirements of subsequent analysis (Figure 1(c)).

As shown in Figures 1(d) and 1(e), there was no significant difference in the alpha diversity between the five groups when assessed using observed species and ACE (*P* > 0.05 for all comparisons between groups).

### 3.3. RDN Reversed the Altered Composition Structure of Gut Microbial Communities Caused by Heart Failure

Beta diversity was analyzed to estimate the extent of variation between gut bacterial profiles of the five groups. PCA, PCOA, and NMDS analyses revealed that the respective distance between the RDN, Nog, and NEP groups and the control group was shorter than the distance between the HF group and the control group.

NMDS statistics showed that the stress was 0.111 (stress <0.2 was used as an acceptable threshold [21]), indicating that NMDS accurately reflected the degree of difference between samples. As shown in Figure 2, most of the HF samples were clustered closely and showed a clear separation from the RDN, Nog, and NEP groups, suggesting that the gut microbiota structure recovered after RDN. The significance of differences was confirmed by the tests of MRPP, AMOVA, ANOSIM, and ADONIS tests (Table 1).

### 3.4. RDN Attenuated Alterations in Fecal Bacterial Abundance Caused by Heart Failure

Figure 3(a) shows that *Firmicutes* and *Bacteroidetes* were the major bacteria in each group at the phylum level. The abundance of *Bacteroidetes* was higher in the HF group (34.56%) than in the control group (24.98%), while *Firmicute* abundance was decreased (59.30% vs. 68.72%). After RDN treatment, this trend reversed. The abundance of *Bacteroidetes* was decreased in the RDN group (18.78%), the Nogo group (12.11%), and the NEP group (18.04%) compared with the HF group (34.56%). The abundance of *Firmicutes* was increased in the RDN group (75.21%), the Nog group (80.03%), and the NEP group (68.91%) compared with the HF group (59.30%). As an indicator of dysbiosis [22], the *Firmicutes/Bacteroidetes* (F/B) ratio of HF rats (1.59) was decreased compared with that of control rats (3.21) and was lower than that of RDN rats (6.20), Nog rats (7.19), and NEP rats (4.42). There was no significant difference between the RDN, Nog, and NEP groups (all *P* > 0.05).  Figure 3(b) also shows that the abundance of *Synergistetes* and *Thermotogae* was increased in the HF group compared with the control group and then decreased in the RDN, Nog, and NEP groups when compared with the HF group.

At the genus level, the HF group possessed decreased abundances of *Lactobacillus* and *Alistipes*, which had potential myocardial protective effects or anti-inflammatory function [23, 24], and increased abundances of *Bacteroides* and *Clostridium*, which were harmful to the myocardium [25], compared with the control group. However, the abundance of *Lactobacillus* and *Alistipes* were increased, and *Bacteroides* and *Clostridium* were decreased in the RDN, Nog, and NEP groups compared to the HF group (Figure 4).

In the Venn diagram (Figure 5(a)), the number of OTUs shared by all groups was 1,076, and the number of unique OTUs were 254 in the HF group, 26 in the control group, 68 in the RDN group, 60 in the Nog group, and 97 in the NEP group. The Venn diagram indicated that the RDN, Nog, and NEP groups shared more OTUs with the control group than the HF group, indicating that RDN attenuated the alterations in fecal bacterial abundance caused by HF.

LEfSe analysis showed the dominant species of the five different groups (linear discriminant analysis >4). The RDN group had increased relative abundances of *Romboutsia*, *Peptostreptococcaceae*, and *Lactobacillus gasseri* (Figures 5(b) and 5(c)). The heat map was constructed and also showed the relative abundance of bacteria in five different groups. The *Faecalibaculum* genus was highly enriched in the RDN group (Figure 5(d)).

### 3.5. RDN Did Not Alter the Composition Structure of Gut Microbial Communities or the Fecal Bacteria Abundance of Normal Rats

As shown in Figure 6, the samples in the Con group and Con + RDN groups were clustered together, suggesting that RDN did not alter the compositional structure of the gut microbial community in normal rats. The abundances of *Firmicutes* ((0.511 ± 0.145) vs. (0.517 ± 0.120); *P*=0.940) and *Bacteroidetes* ((0.324 ± 0.118) vs. (0.273 ± 0.085); *P*=0.449) were not significantly different between the Con and Con + RDN groups. No difference was observed in the *Firmicutes*/*Bacteroidetes* ratio ((1.899 ± 1.280) vs. (1.975 ± 0.483); *P*=0.904) between the two groups. No significant differences were identified between the Con and Con + RDN groups in terms of the abundances of *Alistipes* ((0.001 ± 0.000) vs. (0.004 ± 0.003); *P*=0.070), *Bacteroides* (0.015 (0.001–0.032) vs. 0.036 (0.032–0.056); *P*=0.222), or *Clostridium* ((0.012 ± 0.006) vs. (0.072 ± 0.034); *P*=0.051; Figure 7). These data indicated that RDN could not change the proportion of the gut microbiota in normal rats.

### 3.6. RDN Improved the Predictive Function of the Gut Microbial Population

Tax4Fun analysis allowed us to predict functional pathways potentially affected by the changes in bacteria. The Venn diagram showed that the HF group had 12 unique functional pathways, while there was only one in the control group and zero in the RDN, Nog, and NEP groups (Figure 8(a)). No obvious separation was detected between the RDN, Nog, and NEP groups (Figure 8(b)). As shown in Figure 8(c), bacteria expressing genes associated with amino acid and pyrimidine metabolism were increased in HF rats and decreased after RDN. The functional pathways with statistically significant differences between the HF group and RDN groups are presented in Figure 9. As shown in Figure 9, the KEGG pathway for adenosine triphosphate-binding cassette transport was significantly decreased in the HF group compared with the RDN group. Meanwhile, the tricarboxylic acid cycle pathway, which has central importance to many biochemical pathways, was also significantly increased in the HF group compared with the RDN group. These data indicated that RDN improved the predicted function of the intestinal bacteria.

## 4. Discussion

In this work, the beta diversity was altered in fecal samples of HF rats compared with that of the controls, but these alterations were reversed after RDN treatment. RDN increased the F/B ratio, which was decreased in HF rats. RDN reversed the decreases in *Lactobacillus* and *Alistipes* and the increases in *Bacteroides* and *Clostridium* caused by heart failure. However, no differences were observed between the three groups that underwent RDN. These findings indicated that gut microbiota composition profiles and community structure were altered when heart failure occurred, but these alterations could be reversed by RDN. Reinnervation of renal nerves or inhibition of reinnervation after RDN had no effect on intestinal bacteria.

Consistent with previous studies, our study showed that RDN reduced the plasma concentrations of NT-proBNP in HF rats [12]. There was no substantial difference in NT-proBNP levels between the RDN, Nog, and NEP groups, suggesting that reinnervation of renal nerves after RDN had no impact on cardiac function. PCA, PCOA, and NMDS analyses showed marked separation in HF rats from other groups, indicating that the community structure of intestinal bacteria was altered after heart failure and could be recovered by RDN. The RDN, Nog, and NEP groups clustered together, demonstrating that renal nerve regeneration after RDN did not affect the beta diversity. Since the changes in intestinal bacterial structure are always accompanied by the alternation of gut microbial function, these alterations in the bacterial population and gene expression caused by RDN may benefit cardiac function by influencing the gut microbiota.

In this study, RDN increased the ratio of F/B at the phylum level, which was decreased in rats with HF. It has been reported that products of *Firmicutes* and *Bacteroidetes* have potential impacts on cardiac function. Many bacteria belonging to the *Firmicutes* phylum have butyrate as their primary metabolic end products, which can provide energy to the gut bacteria and the intestinal epithelium, exert local anti-inflammatory effects in the gut wall, and play important roles in maintaining the gut barrier [26]. Mayerhofer et al. found that lower levels of butyrate-producing bacteria were associated with worse outcomes in patients with heart failure [27]. Therefore, *Firmicutes* is beneficial to HF. *Bacteroidetes* are Gram-negative bacteria that can release lipopolysaccharide (LPS) endotoxin. Elevated *Bacteroidetes* in the gut of HF rats may cause an increase in LPS, which contributes to the development of left ventricular dysfunction [28]. Patients with chronic decompensated HF have elevated levels of LPS [29]. In this view, *Bacteroidetes* is harmful to HF. It has been demonstrated that a low F/B ratio was associated with a poor prognosis in HF [30]. In this study, the increased F/B ratio after RDN implied that the role of RDN in improving cardiac function may also by raising the abundance of *Firmicutes* and reducing the abundance of *Bacteroidetes*.

Furthermore, our results showed that some anti-inflammatory bacteria such as *Lactobacillus* and *Alistipes*, which have potential intestinal and myocardial protective roles [23, 24], decreased in HF animals, and increased after RDN, indicating that RDN can influence the abundance of bacteria beneficial to HF. Moreover, the abundance of TMA-producing genera such as *Bacteroides* and *Clostridium* was increased in the HF group and reduced in the RDN group [31]. TMA produced by gut microbes is a precursor of trimethylamine N-oxide (TMAO). TMAO levels were directly correlated with the severity of HF and unfavorable outcomes in HF patients [32]. RDN affected the bacteria abundance of HF rats. These data suggested that RDN could also improve cardiac function by promoting the growth of beneficial bacteria and inhibiting the proliferation of bacteria harmful to HF. In this view, the altered gut microbiota composition profiles and community structure when heart failure occurs can be reversed by RDN. It remains unknown whether RDN can change the proportion of the gut microbiota in normal rats. However, our study showed that the composition and diversity of the gut microbiota in the Con and Con + RDN groups did not differ, which indicated that RDN did not change the proportion of the gut microbiota in normal rats. Therefore, RDN may improve cardiac function by influencing intestinal bacteria.

Adenosine triphosphate-binding cassette (ABC) transport involves transmembrane proteins localized in many tissues, including the heart and intestine. ABC transport in the heart can exert a protective effect against chemical injury or oxidative stress, and many transporters have roles in controlling the absorption and distribution of endogenous substrates or xenobiotics in the intestine [33]. In our study, KEGG results showed that ABC transport was significantly increased in the RDN group compared with the HF group, suggesting that RDN may also affect metabolism in heart failure.

Increased sympathetic activity to the gut could lead to an imbalance of short-chain fatty-acid-producing bacteria and stimulate the growth of a range of bacterial species [8, 34]. The role of RDN in mitigating aberrant intestinal bacteria in this study may be related to its function in reducing intestinal sympathetic activity. In addition, our study showed that inhibition reinnervation after RDN did not affect either cardiac function or the gut microbiota. Perhaps the regenerated nerve fibers were not functional [35] and thus had no effect on gut bacteria, even if anatomic reinnervation was present.

Several limitations should be discussed. First, gut neural activity in rats after RDN was not recorded. The degree of decrease in the intestinal sympathetic nerve activity was not clear. The relationship between intestinal sympathetic nerve activity and gut microbiota remains to be determined, and it is necessary to validate this work. Second, some important bacterial products related to HF, such as TMAO, were not detected. Bacterial products may be more important to HF than bacteria themselves.

## 5. Conclusions

RDN recovered the altered composition structure of gut microbial communities caused by HF and increased the F/B ratio, which was decreased in HF rats. RDN also increased the abundances of some beneficial bacteria to HF, such as *Lactobacillus* and *Alistipes*, and reduced the abundances of some harmful bacteria such as *Bacteroides* and *Clostridium*. However, no differences in the changes in the gut microbiome were observed between RDN rats regardless of whether they were administered an inhibitor of axonal regeneration or its antagonist. This study showed that RDN could reverse the abnormal changes in the gut microbiome in HF. The beneficial effect of RDN on cardiac function may also be mediated by influencing intestinal bacteria. Inhibition of reinnervation after RDN did not affect intestinal bacteria.

## Figures and Tables

**Figure 1:** Schematic diagram of the study and the influence of RDN on plasma N-terminal prohormone brain natriuretic peptide (NT-proBNP) levels and alpha diversity of the gut microbiome. (a) Schematic diagram of the study. (b) Plasm NT-proBNP levels of the control group, the HF group, the RDN group, the Nog group, and the NEP group (^*∗*^*P* < 0.05 vs. the HF group). (c) Rarefaction diversity of different samples based on observed species number. The sequencing depth is given on the *x*-axis, while the *y*-axis shows the corresponding operational taxonomic units (OTUs). (d, e) Alpha diversity for various groups based on observed species and abundance coverage estimator (ACE). No significant differences were found between the five groups (*P* > 0.05).

**Figure 2:** RDN reversed the altered composition structure of gut microbial communities caused by heart failure: (a) PCoA based on the unweighted Unifrac distance, (b) principal component analysis (PCA), and (c) nonmetric multidimensional scaling (NMDS) analysis (stress = 0.111) of bacterial population structure. Dots of different colors represent different samples from the control group (red), the HF group (blue), the RDN group (green), the Nog group (yellow), and the NEP group (purple). As presented in the figure, samples from the control group, the RDN group, the Nog group, and the NEP group clustered together and kept away from the HF group.

**Figure 3:** RDN attenuated alterations in fecal bacteria abundance at the phylum level caused by HF. (a) Relative abundance distribution of the top 10 bacteria at the phylum level. The HF group had the highest abundance of *Bacteroidetes* and the lowest abundance of *Firmicutes*. (b) Metastats analysis of differences at the phylum level for *Firmicutes*, *Bacteroidetes*, *Actinobacteria*, *Chloroflexi*, *Synergistetes*, and *Thermotogae* (^*∗*^*P* < 0.05 and ^*∗∗*^*P* < 0.01).

**Figure 4:** RDN attenuated alterations in fecal bacteria abundance at the genus level caused by HF. (a) Relative abundance distribution of the top 10 bacteria at the genus level. Compared with other groups, the HF group had higher abundance of *Bacteroides* and lower abundance of *Lactobacillus*. (b) Metastats analysis of differences at the genus level for *Clostridium*, *Bacteroidetes*, *Lactobacillus*, and *Alistipes*. ^*∗*^*P* < 0.05 and ^*∗∗*^*P* < 0.01.

**Figure 5:** The results of Venn diagram, LEfSe analysis, and heat map analysis. (a) Venn diagrams and unique operational taxonomic units (OTUs) among the intestinal bacterial communities of the control, HF, RDN, Nog, and NEP groups. (b) The results of linear discriminant analysis effect size (LEfSe). The histogram of the linear discriminant analysis (LDA) score showed the biomarkers with statistics in the control (red), HF (green), RDN (purple), Nog (yellow), and NEP (blue) groups (LDA score ≥4.0). The degree to which species exerted an influence is expressed by the length of the bar in the histogram. (c) Taxonomic cladogram obtained from LEfSe. Taxa meeting a linear discriminant analysis significance threshold >4 are shown (c: class level; f: family level; g: genus level; o: order level; and p: phylum level). Biomarkers were colored by different groups (yellow represented nonsignificant, red indicated the control group, green indicated the HF group, purple indicated the RDN group, yellow indicated the Nog group, and blue indicated the NEP group). Each circle's diameter was proportional to the taxonomic abundance. (d) Heat map of the top 35 genera of relative abundance of rats gut microbes from the control, HF, RDN, Nog, and NEP groups. The relative abundance of different genera was presented with a color gradient from deep blue (low abundance) to deep red (high abundance).

**Figure 6:** RDN did not alter the compositional structure of the gut microbial community in normal rats: (a) PCoA, (b) PCA, and (c) NMDS analyses of bacterial population structure. The colored dots in the panel represented different samples (Con: normal rats received sham RDN; Con + RDN: normal rats received RDN operation).

**Figure 7:** RDN did not alter the fecal bacterial abundance of normal rats at the phylum and genus levels. (a) Relative abundance distribution of the top 10 bacteria at the phylum level of the Con and Con + RDN groups. Comparison of the *Firmicutes/Bacteroidetes* ratio (b) and the abundances of *Firmicutes* (c) and *Bacteroidetes* (d) between the Con and Con + RDN groups. Comparison of the abundances of *Alistipes* (e), *Bacteroides* (f), and *Clostridium* (g) between the Con and Con + RDN groups. ^*∗*^*P* < 0.05.

**Figure 8:** Functional and pathway enrichment analyses of amplicon sequencing results using the Kyoto Encyclopedia of Genes and Genomes (KEGG) database. (a) Venn diagrams and unique pathways among the intestinal bacterial communities of rats in the control, HF, Nog, and NEP groups. (b) Principal component analysis (PCA) plot showing the first two principal components of the third level KEGG functions. The five groups were not separated well. PC1: the first principal coordinate; PC2: the second principal coordinate. (c) The third level of the KEGG pathway was shown in the heatmap. Relative abundances of different pathways was presented with a color gradient from deep blue (low abundance) to deep red (high abundance).

**Figure 9:** Distinct Kyoto Encyclopedia of Genes and Genomes (KEGG) functions in the HF group (yellow) and the RDN group (blue). *P* < 0.05 as per *t* test.

**Table 1:** Significance tests on community structures between groups with MRPP, AMOVA, ANOSIM, and ADONIS tests.

Groups	MRPP		AMOVA	ANOSIM		ADONIS	
	*A*	*P*	*P*	*R*	*P*	*R* ^2^	*P*
Control vs. HF	0.04	**0.026**	0.095	0.42	**0.012**	0.17	**0.020**
Control vs. RDN	−0.00	0.471	0.603	0.04	0.536	0.10	0.567
Control vs. NEP	0.05	0.056	0.348	0.17	0.16	0.18	0.084
Control vs. Nog	0.02	0.148	0.071	0.15	0.167	0.13	0.168
HF vs. RDN	0.07	**0.003**	**0.015**	0.48	**0.006**	0.21	**0.008**
HF vs. NEP	0.09	**0.002**	**0.010**	0.63	**0.001**	0.24	**0.001**
HF vs. Nog	0.10	**0.002**	**0.001**	0.61	**0.002**	0.25	**0.001**
RDN vs. NEP	0.03	0.077	0.315	0.14	0.167	0.14	0.126
RDN vs. Nog	−0.00	0.433	0.585	0.05	0.279	0.08	0.540
NEP vs. Nog	0.05	**0.008**	0.170	0.24	**0.026**	0.16	**0.015**

Bold values indicate statistical significance (*P* < 0.005). “*A*” values in the MRPP test greater than 0 indicated that the intergroup difference is greater than the intragroup difference, but “*A*” values less than 0 indicated that the intragroup difference is greater than intergroup difference. In the ANOSIM test, *R* > 0 indicated that the differences between the groups were larger than the differences within the groups. The larger *R*^2^ value in the ADONIS test indicated a better explanation for the classified difference. MRPP: multiresponse replacement process; AMOVA: analysis of molecular variance; ANOSIM: analysis of similarity; ADONIS: analysis of distance matrices.

## Data Availability

The data sets used and/or analyzed during the current study are available from the corresponding author on reasonable request.
